The article "Factors That Affect Maternal Mortality in Rwanda: A Comparative Study with India and Bangladesh" was retracted in 2023. Reasons: signs of a paper mill; suspected computer-generated content; unreliable results or conclusions; lack of ethics approval or compliance.

# Factors That Affect Maternal Mortality in Rwanda: A Comparative Study with India and Bangladesh

**DOI:** 10.1155/2022/1940188

**Published:** 2022-04-09

**Authors:** Mugenzi Patrick, Muhammad Sami uz Zaman, Ghazala Afzal, Minhas Mahsud, Mumuni Napari Hanifatu

**Affiliations:** ^1^Beijing University of Aeronautics & Astronautics (BUAA), Beijing, China; ^2^Pak Red Crescent Teaching Hospital Dinanath, Lahore, Pakistan; ^3^National University of Sciences and Technology Islamabad, Pakistan; ^4^University for Development Studies, Ghana

## Abstract

Healthcare sector is one of the most pivotal pillars of the administrative setup of a country. It addresses one of the most important dilemmas that countries have to face: provision of quality healthcare to public in affordable prices. Africa lags behind in many health indicators. One of the contemporary health issues faced by countries, especially for those in sub-Sahara countries, is maternal mortality rate (MMR). It has had a significant part to play in the social conditions of the population and needs immediate attention. In spite of many years of civil war and the terrible genocide in the mid-1990s, as of late, Rwanda is showing signs of improvement in healthcare sector. This research is aimed at studying the current state of maternal mortality rate in Rwanda and the factors behind its performance, in a comparative study with India and Bangladesh for a cross-section of time mainly between 1990 and 2015. After a literature review, pivotal indicators that affect healthcare are shortlisted and a comparative analysis of the three countries is made on the basis of these indicators. A regression is run between historical MMR data and these indicators. A directly significant relationship is found between MMR and healthcare expenditure per capita and government commitment to health, closely followed by female literacy and healthcare infrastructure.

## 1. Introduction

In spite of many years of civil war and the terrible genocide in the mid-1990s which crushed the nation's health framework, as of late, Rwanda has been a model of enhancing access to maternal human services. Rwanda has a big poverty problem, and the nation has an expansive rustic populace, influencing access to healthcare facilities, especially for women. Unintended pregnancies lead to prebirth complications and risky premature births, which, coupled with strained assets at the provincial and regional levels, adds to maternal dismalness and mortality.

However, the Rwandan government has made enhancing family planning services a national priority. Working with the World Health Organization, the Rwandan Ministry of Health has organized contracting and preparing health workers to give family planning instruction, family counseling, and such services to the men and women throughout the nation. Thus, Rwanda's maternal mortality rate (MMR) fell by a lot recently. The maternal mortality rate in Rwanda has seen a huge drop from 750 in 2005 (DHS) to 540 in year 2008 and under 400 as indicated by Health Management Information System (HMIS: 2010) and under 300 (RDHS) in 2015. Deliveries by Health Workers expanded from 38 percent in 2005 (DHS) to 52 percent in 2007 (DHS 2007) and 63.5 percent in 2010 (HMIS). The maternal mortality rate has fallen as of late, but is still high. Enhanced healthcare reconnaissance and responsibility have assumed a huge part in diminishing the MMR and expanding the quantity and quality of assisted deliveries in Rwanda. Enhanced surveillance has enabled Rwanda's Ministry of Health to better track the reasons for maternal deaths all through the nation, bringing about more focused approaches and techniques to counter the issues. Some important factors comprise the high percentage of births that take place without skilled assistance (52%) and the lesser utilization of family planning and basic obstetrics care (CPR: 27%).

The article "Factors That Affect Maternal Mortality in Rwanda: A Comparative Study with India and Bangladesh" was retracted in 2023. Reasons: signs of a paper mill; suspected computer-generated content; unreliable results or conclusions; lack of ethics approval or compliance.

UNFPA is another organization that has been working in these fields in Rwanda since 1975. From that time on, it has been effective in progressing and supporting reproductive health and rights, gender, population, and development in Rwanda at both the focal and decentralized levels. According to UNFPA, roughly 800 women pass away from preventable issues during pregnancy and childbirth, 99% of all maternal deaths happen in developing nations, and they are to a great extent preventable [1]. The maternal mortality proportion in developing nations is 240 for each 100,000 births versus 16 for each 100,000 in developed nations. There are substantial incongruities between nations in MMR, with some nations having a very high maternal mortality rate of 1,000 or more per 100,000 live births; more than half of all maternal deaths happen in sub-Saharan Africa and just about 33 percent happen in South Asia [1]. The WHO classifies limited access to services, poverty, information lack, and a dearth of cultural practices in health as main causes of variances in MMR. The strategy reports on maternal mortality only from time to time demonstrate trainings as a reason, and the research has almost nothing to say with regard to the connection between maternal mortality and training. All things considered, it could be said that a positive relationship among instruction and different pointers of well-being exists. A viewpoint suggests that people who are more educated care for and look for medical care more often than those who are less literate [2–4]. This is predictable with the viability that education helps procuring and handling significant data [5, 6]. Education may likewise impact health through its effect on pay but not the same as that of income [4, 6]. However, the studies [7, 8] underscore the influential role of education in reducing maternal mortality. Generally, this study is aimed at studying the data on maternal mortality and how it is affected by some of the selected health indicators, including education, as shall be seen later.

The article "Factors That Affect Maternal Mortality in Rwanda: A Comparative Study with India and Bangladesh" was retracted in 2023. Reasons: signs of a paper mill; suspected computer-generated content; unreliable results or conclusions; lack of ethics approval or compliance.

In the Rwandan context, MMR has had a significant part to play in the social conditions of the population. The issue of MMR is not being given serious thought and that is why it needs the immediate attention for the betterment of healthcare provision to adult Rwandan females. If we look on the global scale, sustained health plans, government commitment and foreign aid for health programs have shown meaningful results all across the globe in reducing MMR. Some countries like Bangladesh, Nepal, India, and Honduras have taken concrete steps and performed really well, indicating that if the vision is correct, things shall and do get better. It is important that we learn from the past and not repeat the same mistakes. A previous research by a study [9] evidently points out a relationship between increased maternal survival and the need of education among other factors. It is of utmost importance that these factors are continually investigated especially for all developing countries, not only Rwanda, so as to pinpoint where things are going wrong and why. This research undergoes some limitations; specifically, few empirical researches have analyzed the factors behind improved maternal mortality rate.

This study intends to investigate some facets of Rwandan economy, society, social set-up, governance, and the relevant infrastructure in place and their contributions to the health of an average Rwandan woman. In this regard, this research is aimed at studying the current state of maternal mortality rate in Rwanda and the factors behind its performance, in a comparative study with India and Bangladesh which have been able to perform very well in decreasing MMR for the adult female populations. The choice of variables used in this study resulted from the review of the literature and as a result pivotal indicators or factors that affect healthcare are shortlisted, and we have identified country's economy represented by GDP per capita, health expenditure per capita, government commitment, female literacy rate, healthcare infrastructure and improvement in sanitation, sanitation facilities, and presence of nurses and midwives as commendable studies recommend these factors as building blocks contributing to maternal health [10–14].

The article "Factors That Affect Maternal Mortality in Rwanda: A Comparative Study with India and Bangladesh" was retracted in 2023. Reasons: signs of a paper mill; suspected computer-generated content; unreliable results or conclusions; lack of ethics approval or compliance.

## 2. Literature Review

### 2.1. Definition of Maternal Mortality

As per the United Nations Maternal Mortality Estimation Inter-office Group, which comprises delegates from the World Health Organization (WHO), United Nations Children's Fund (UNICEF), the United Nations Population Fund (UNFPA), United Nations Population Division, the World Bank, and widely acclaimed academicians, maternal demise is the passing of a woman while pregnant or within 42 days after delivery of a baby, regardless of the term and the site of the pregnancy, from any reason identified with or exasperated by the pregnancy or its administration, not from inadvertent or accidental causes [15]. Maternal death is measured by some indicators of MMR such as the maternal mortality rate, maternal death lifetime risk, and maternal deaths among deaths of women of age of reproduction (PM).

### 2.2. Factors Determining Maternal Mortality

Variables that determine maternal death can either be direct or indirect. For the most part, direct causes of maternal demise occur as the after effect of an issue of the pregnancy, delivery, or mismanagement of either of these; indirect maternal demise is a pregnancy-related death in a patient with a prior or recently created health issue not related to pregnancy. Fatalities, during but not related to pregnancy, are namely accidental, incidental, or nonobstetrical maternal deaths. As expressed by a study [16] “Make Each Mother and Child Count,” the major direct reasons for maternal deaths are serious blood-loss/hemorrhage (25 percent), infections (13 percent), hazardous abortions (13 percent), eclampsia (12 percent), deterred labor (8 percent), other direct causes (8 percent), and indirect causes (20 percent). Indirect causes are malaria, anemia, HIV/AIDS, and cardiovascular sickness, all of which may confound pregnancy or be exasperated by it. Socioeconomic factors, like age, access to resources, and salary level, are noteworthy pointers of maternal demise. Young mothers confront higher dangers of complexities and demise during pregnancy than older mothers, who have higher dangers of creating postpartum hemorrhage, puerperal-endometriosis, operative vaginal delivery, episiotomy, low birth weight, preterm delivery, and small-for-gestational-age babies, all of which can prompt demise of the mother. Basic care and family support influences results for mothers. Besides, social disservice and social seclusion unfavorably influence maternal well-being, which can prompt increments in maternal demise. Also, absence of access to skilled Medicare during labor, trouble of movement to the closest center to get appropriate care, number of earlier births, absence of prebirth therapeutic care, and poor health framework all add to maternal mortality. Another investigation [17] states that unsafe abortion is another significant reason for maternal passing. As per the World Health Organization, one mother passes from inconveniences emerging from perilous premature births every eight minutes from intricacies arising from hemorrhage, infection, sepsis, and genital trauma. Universally, preventable demise from improperly performed procedures constitutes 13% of maternal mortality, and at least 25% in a few nations where maternal mortality from different causes is moderately low, making unsafe abortion the biggest reason for maternal mortality.

The article "Factors That Affect Maternal Mortality in Rwanda: A Comparative Study with India and Bangladesh" was retracted in 2023. Reasons: signs of a paper mill; suspected computer-generated content; unreliable results or conclusions; lack of ethics approval or compliance.

Another study [18] considerably suggested that maternal mortality is significantly related to women education which is also influenced by various aspects including geographical, economic, religious, sociocultural, legal, and political issues.

### 2.3. Measurement of Maternal Death

The four measures of maternal demise are maternal mortality proportion (MMP), maternal mortality ratio (MMR), lifetime risk of maternal demise, and extent of maternal demise among deaths of Women of Reproductive Years (PM). Maternal mortality proportion (MMP) is the proportion of the quantity of maternal deaths amid a given time period per 100,000 live births over the same time period. Maternal mortality rate (MMR) is the quantity of maternal deaths in a populace isolated by the quantity of women of regenerative age, normally measured per 1,000 women. Lifetime risk of maternal death alludes to the likelihood that a 15-year-old female will pass on in the end from a maternal reason on the off chance that she encounters, all through her lifetime, the dangers of maternal demise, and the general levels of fertility and mortality that are watched for a given population. This rate can be determined utilizing either the maternal mortality proportion (MMP) or the maternal death rate (MMR). Finally, the extent of maternal` deaths among deaths of women of reproductive age (PM) is the quantity of maternal deaths in a given day and age partitioned by the aggregate demises among women between the ages of 15 and 49 years. This study employs and uses the MMR for countries in comparison and analysis/results. Ways to deal with estimating maternal mortality incorporate civil registration framework, household reviews, census, Reproductive Age Mortality Studies (RAMOS), and verbal autopsies.

### 2.4. The State of Maternal Mortality in Developing Countries

At the end of the last century, sub-Saharan Africa still had high maternal mortality and death rates, with the objectives of safe parenthood eluding numerous administrations. The Program of Action of the International Conference on Population and Development, 1994, and the Fourth World Conference on Women, 1995, were made to handle these issues. These projects drew extraordinary regard for reproductive well-being and rights and to sexual orientation value and equality. The scourge of the Human Immunodeficiency Virus (HIV) and Acquired Immune Deficiency Syndrome (AIDS) desolated the population and left in its wake untold demolition in the statistic, monetary, and social circles (UN, 2003). Statistics from the most recent decade are in sharp contrast to those in the 1980s, while diminishing infant, young, and grown-up death rates and maternal mortality proportions (MMP) were prompting expanding life expectancy and better health status for women in the locale.

The article "Factors That Affect Maternal Mortality in Rwanda: A Comparative Study with India and Bangladesh" was retracted in 2023. Reasons: signs of a paper mill; suspected computer-generated content; unreliable results or conclusions; lack of ethics approval or compliance.

Bangladesh is a great instance of a low and middle wage nation accomplishing the improbable, which numerous others neglected to do. It lessened its maternal mortality by 66 percent in the period of 1990 and 2010; the decrease was 40 percent from 2001 and 2010 alone. These were accomplished by bringing down the maternal mortality rate (the quantity of maternal deaths per 100,000 Live Births) from 574 to fewer than 200 in the period from 1990 to 2010. The diminishment was significant for eight years (1990 to 1998), as MMR diminished from 574 to 322 for each 100,000 live births. According to the 2012 WHO statistics, the normal yearly rate of this decrease was 5.9 percent in a period from 1990 to 2010, which is more than the Millennium Development Goal 5 focus of 5.5 percent or more. What is all, the more astonishing is that the diminishment in MMR (maternal deaths per 100,000 live births) was nearly the same in both the urban and provincial territories. At the present rate, Bangladesh is well on its way in achieving the MDG 5 focus of 143 for each 100,000 live births an entire year before its designated time. Another example is India which has been able to excessively lessened maternal mortality by 65 percent from 569 to 190 for each 100,000 live births from 1990 to 2013. However, with 4.5 percent annual decrease in MMR, India might just miss the MDG 5 focus of 5.5 percent or more abatement rate before 2015. Be that as it may, the execution by India has been excellent from that point onward. [19].

#### 2.4.1. Pivotal Success Factors for MMR Decrease

A study [20] exhibited that the decline in maternal mortality was given due importance in mid-to-late 19^th^ century in northwestern Europe (Sweden, Netherland, Denmark and Norway). The concept of MMR expanded later in Britain and USA, moving in to lesser developed countries as a pivotal factor of maternal well-being. Today, maternal health is an important measure of national health. How did Bangladesh, one of the poorest nations on the planet with the most population density and where 75 percent of the populace lives in rural areas, rapidly accomplish MMR decrease? Furthermore, how did India oversee such a change? It is a difficult inquiry to reply to. As indicated by [21], the status and value of women have definitely improved. They are more literate in ways of the world. Oppression of women has descended too.

The article "Factors That Affect Maternal Mortality in Rwanda: A Comparative Study with India and Bangladesh" was retracted in 2023. Reasons: signs of a paper mill; suspected computer-generated content; unreliable results or conclusions; lack of ethics approval or compliance.

Between 1930 and 1995, Malaysia and Sri Lanka succeeded, through similar means, in diminishing their MMRs significantly every 6-12 years down to fewer than 50 for each 100,000 live- births by 1995. In the 1930s, Malaysia, notwithstanding gloating a moderately solid economy, and Sri Lanka, a low-salary nation with extraordinarily large amounts of female education, were both tormented by MMRs of more than 500 for every 100,000 Live Births and more than 2000 for every 100,000 Live-Births, respectively. Understanding the overwhelming impact of the poor providence of maternal health on national development and advancement, the two nations actualized exhaustive national systems to diminish maternal mortality. Four key parts added to the achievement of both national projects: extensive strengthening of human development programs (i.e., education, infrastructure, sanitation, and health frameworks) particularly in poor and underserved territories; noteworthy interests in enhanced maternal well-being administrations, enhanced access to proficient nurses and midwives; and progressing political help will decrease MMR. Outstandingly, concurrent with maternal mortality decay amid this period, Sri Lanka additionally diminished its TFR from 5 to 2.2 live births per woman in age of conception and Malaysia from 6.3 to 3.4 live births per women of reproductive age. Supported by great political will and dynamic political bodies focused on decreasing Maternal Mortality in both nations, infrastructure investments, rural health facilities, and human resources empowered the administrations of Sri Lanka and Malaysia to help underprivileged masses [22]. Access to essential health centers quickly expanded. Other human advancement programs, for example, adult education activities and maternal well-being efforts, prompted enhanced information and comprehension of the significance of skilled attendance during childbirth. Surprisingly, neither one of the countries spent in excess of 3 percent of its GDP on health, uniquely lower than different nations of a comparative monetary standing. Against this background, both Sri Lanka and Malaysia set out a remarkable journey to end MMR. These projects prepared nurses and midwives to deal with essential complications in childbirth, connected them to the formal healthcare framework and empowered coordinated effort with doctor's facilities and focus on health. With the advantage of a recently expanded status inside networks, naturally prepared nurses and midwives were sent in provincial areas [23]. Family planning inputs would allow for considerable reductions in maternal deaths worldwide, with the authors estimating that the equivalent of 44% of maternal deaths in 2008 were averted due to contraceptive use and that meeting unmet demand for family planning could prevent a further 29% of maternal deaths [21].

The article "Factors That Affect Maternal Mortality in Rwanda: A Comparative Study with India and Bangladesh" was retracted in 2023. Reasons: signs of a paper mill; suspected computer-generated content; unreliable results or conclusions; lack of ethics approval or compliance.

A research study suggested that skilled attendance at childbirth is effectively linked to decrease in maternal mortality in Sweden. On the other hand, the researches that have been done in USA and Netherlands in the 1900s attributed a decline in maternal mortality to the changes in population age and parity [24].

In this study, we shall take a special look at the four human development factors (i.e., education, infrastructure, sanitation, and health frameworks) recommended in many studies [10–14], which are pivotal for success in decreasing MMR substantially. A comparison shall be made between countries of India and Bangladesh with Rwanda, and analysis shall be done, to see how Rwanda fares against these two.

## 3. Design and Data Analysis

A detailed cross-sectional comparative study between Rwanda and the South East Asian countries of Bangladesh and India shall be done. These are countries that have been able to effectively achieve their MDG 5 goals, especially in maternal mortality, as per the WHO guidelines. The studies shall focus on the most important points relevant to this study as mentioned in the literature and shall elaborate how; over time, these countries have fared. This study [25] defines a source of data as one of the materials the researcher utilize for collecting information during investigation. The study has incorporated data from comprehensive country reports by the UN, World Health Organization (WHO), DHS, UNICEF, World Bank, and other international and national agencies with published data. Historical data taken only from commendable sources from different cross-sections of time (mainly between 1990 and 2015) are used in the analysis. A regression shall be run on the basis of this data, and results shall be achieved.

### 3.1. Maternal Mortality (MMR)

The indicator MMR, that measures number of annual maternal deaths as a fraction of 100,000 live births of a country in the same period, is the most important feature. An optimum value to be achieved for it is 143, which shall be used as a benchmark. The comparison is in Figure 1. Figure 1 as per SDGs shows that the MMR curves for India and Bangladesh are pretty linear, starting around the 600 mark in 1990 and decreasing somehow linearly up till the latest data line, which shows the MMR to have dropped to the 170/100,000 maternal deaths around 2015 for India and Bangladesh. According to expert forecasts, Bangladesh is being tipped to achieve the desired mark fairly soon now in 2020, whereas India is expected to miss it by a narrow margin. Rwanda, after a qualitative forecast analysis depending upon historical data, is tipped to achieve this number by 2025. The data for Rwanda has been nothing short of a revelation which saw MMR rates start from as high as 1300/100,000 in 1990 and then almost becoming half from 1020 in 2000 to 567 in 2005. It has since been decreasing at a rate faster than that of either Bangladesh or India, due to efficient government policies and a healthcare system designed for those who cannot afford it. It has been because of these efforts the MMR for Rwanda is being predicted to fall below that of India and Bangladesh, a huge result. The rates after 2020 are forecasts based upon past data.

The article "Factors That Affect Maternal Mortality in Rwanda: A Comparative Study with India and Bangladesh" was retracted in 2023. Reasons: signs of a paper mill; suspected computer-generated content; unreliable results or conclusions; lack of ethics approval or compliance.

### 3.2. GDP per Capita Data

To measure the rate of economic wealth per person for all three countries (gross domestic product divided by midyear population as per World Bank), following is a comparative study of GDP/capita (in USD) of the countries over a period starting from 1990, although data from commendable sources is from 2000 onwards to 2017.

Figure 2 shows how India has been able to accumulate its wealth and is fast becoming an economic power to reckon with after the turn of the century, and the economic growth has been constant, with some hiccups in the middle. A steady increase since 2003 reached a record when it was doubled in 2009, and it kept on increasing at a steady rate, reaching a peak of around 1900 USD in 2017. For Bangladesh, more than a 100 percent increase was seen between 2003 and 2011 with the amount increasing from around 950 USD/person to 1500 USD/person, a net increase on more than 50 percent, between 2013 and 2017, a sign of why things have been turning around in Bangladesh especially in the health sector. Rwanda is not a country with such big amounts of economy to boast, but with the slump in the early 2000s, the economy of the country is at a steady rise with the government investing more and more. This rate though somehow stalled as of late.

### 3.3. Health Expenditure per Capita

A very important factor of those mentioned before has been the government commitment to making health a priority in policy setting for country and appreciable budget allocation to improving healthcare.  Figure 3 shows a trend of how the three governments have fared in health expenditure per capita in US dollars from 2000 to 2015. The results show a steady increase in the health expenditure data for all three countries, which is instrumental in improving the outlook of healthcare provision. Bangladesh has seen a steady increase in health expenditure per capita doubling the rate of 15.4 USD per capita from 2008 to around 32 USD according to data. The same for India has also been seen to rise at a fast rate, picking up in 2009 to around 34 and soaring to 63 USD per capita according to data. Rwanda has shown the most improvement, whereby the per capita spending increased exponentially after 2002 and kept on increasing. The per capita funding doubled in a single year 8.6 USD per capita in 2002 to more than 16 USD in 2003 and reaching a record high of 59 USD in 2014. A good explanation of these phenomena can be attributed to the health and Medicare aid provided to Rwanda from external sources and other countries, which currently fund 53 percent of all healthcare resources of Rwanda.

The article "Factors That Affect Maternal Mortality in Rwanda: A Comparative Study with India and Bangladesh" was retracted in 2023. Reasons: signs of a paper mill; suspected computer-generated content; unreliable results or conclusions; lack of ethics approval or compliance.

### 3.4. Government Commitment (Monetary)

An important indicator when talking about health is the government commitment. The budget committed to the cause of health is a direct indicator of how seriously a country wants to address this issue. A comparison for the three countries is done, and Figure 4 rightly presents the results from 1995 to 2012.

Rwanda has especially surpassed both India and Bangladesh due to appreciable foreign funding for health sector, which is bringing about major changes in the way things are shaping up. Especially in the 2000s the commitment to health has been solid, with the record high of 16% for Rwanda in 2003 and then a whopping 23% in 2006. The number for Rwanda presented here is in 2012 at around 24%. The government commitment trend remains somehow linear for India and Bangladesh, standing at 9% and 8%, respectively.

### 3.5. Female Literacy Rate

Another important indicator especially for this specific research is the female education. It is a very relevant indicator to give us an insight into how lives can be saved through education. The following comparison shows the numbers for adult female literacy rates in these countries in Figure 5 with commendable data from 1991 to 2015.

Bangladesh has shown a very optimum improvement in the literacy rate when in 1991 it was recorded to be around 26 percent and it went up to around 70% in 2015, a figure which is commendable. The percentage for India was 63% in 2015, which is appreciable, but the rise has been steady, starting from 34 percent in 1991. Rwanda has also shown a somehow steady rise in adult female literacy rate, going up from 37% in 1991 to around 67% in 2015.

The article "Factors That Affect Maternal Mortality in Rwanda: A Comparative Study with India and Bangladesh" was retracted in 2023. Reasons: signs of a paper mill; suspected computer-generated content; unreliable results or conclusions; lack of ethics approval or compliance.

### 3.6. Healthcare Infrastructure and Improvement in Sanitation

A prime factor that is being measured is the investment in healthcare infrastructure by the government and improvement in access to sanitation facilities.  Figure 6 presents a comparative study between the three countries in terms of healthcare infrastructure (measured primarily by the increase in hospital beds per person and number of nurses and midwives (which effects MMR directly) with data only from the most commendable sources (2005-2011)). The figure portrays the number of hospital beds per 1000 people in three countries Bangladesh, India, and Rwanda. It reveals that there is an upward slope in the number of hospital beds in both countries Rwanda and Bangladesh, while India presents a steady decrease between 2005 and 2006 and a sharp drop of hospital beds after 2006. In general, Rwanda has a high ratio of hospital beds per 1000 people, though there is no global cutoff metric.

### 3.7. Sanitation Facilities

Governments of the three countries Rwanda, Bangladesh, and India have endeavored to improve health through providing better sanitation facilities to the public.  Figure 7 presents the comparison of percentage of population with improved access to sanitation facilities in those countries from 1990 to 2018. In the period between 1990 and 1999, Bangladesh had a higher percentage compared with others nearly 40%; however, from 2000 onwards, Rwanda rose sharply in numbers and hit approximately 45% of its population that have access to sanitation facilities and increased the slope thereafter. Finally, from 2010 onwards, Rwanda shows improvement with more than 75% of population who access sanitation facilities; more generally in all the period, India exhibits a small number less than 40% of population who have access to sanitation.

### 3.8. Nurses and Midwives

The ratio of nurses and midwives is among the factors that are highly considered in analyzing the progress of health sector. Therefore, following Figure 8 compares Rwanda, Bangladesh, and India in respect of number of nurses and midwives per 1000 people in the period between 2004 and 2015. At first glance, India clearly exhibits a high number since 2004 and increased slightly until 2010. More interestingly from 2010, the ratio increased sharply close to hit the global target of 2.3 which is presumed to be attained soon. In addition, Rwanda also shows an increase in the period of 2005 to 2008 and recently between 2010 and 2015, and we can predict that if the number continues to grow at this rate Rwanda will hit the global target by 2050 [2].

The article "Factors That Affect Maternal Mortality in Rwanda: A Comparative Study with India and Bangladesh" was retracted in 2023. Reasons: signs of a paper mill; suspected computer-generated content; unreliable results or conclusions; lack of ethics approval or compliance.

#### 3.8.1. Model: Regression Analysis

Now that we have had a cursory look at the data, this paper utilizes simple regression model in estimating the factors that affect maternal mortality in Rwanda. The software used is R. The model is specified as follows:

(1) $$\begin{array}{c} {\text{MMR}}_{t}=\beta_{0}+\beta_{1}X_{t}+\varepsilon_{t}. \end{array}$$

The above general specification model is divided into six simple regression models, with each model account variables such as female literacy rate (FLR), budget committed to health (BCH), health expenditure (HE), nurses and midwives (NMd), and sanitation and facilities (SF) as grouped in one single variable *X*_*t*_ in equation (1). The dependent variable MMR stands for maternal mortality rate. This research uses published commendable data from international sources spanning from a cross-section of time.

From the results of regression presented in Table 1, a positively significant relationship is found between MMR and healthcare expenditure per capita. The test indicates that if there is an increase of 1 unit of percentage of healthcare expenditure per capita by the government (measured in USD), it can save as many as 17 female Rwandan lives. As an example, as the latest healthcare expenditure per capita is 67.3 USD for Rwanda for one person, a unit increase of 1% in this amount per person might be able to save 17 female lives who can conceive (Model 4). This is a very significant statistic. Budget commitment to health is also significantly related, whereby the data reveals that if 2 units of the measurement are increased in allocation of healthcare budget, it can save one female Rwandan life (2∗0.5035 = 1.07 lives, model 3). Female literacy (model 2) and sanitation infrastructure (model 6) also demonstrate significant trends towards MMR (Table 1).

## 4. Conclusion and Recommendation

After presenting all of these results, the conclusions in a nutshell and an analysis of how Rwanda is progressing in the quest to decrease MMR shall be presented. The MMR rate for Rwanda has gone down at an appreciable extent, and it is ably competing with other countries, which have been doing well in this regard. At the present rate, Rwanda shall also be listed in countries that have successfully battled with maternal mortality, especially among those of sub-Saharan Africa where it still remains a big issue. Rwanda is on the way to a steady recovery after a slump in the early 2000s, as the government is also investing more towards health as it has now a very impressive share in the GDP per capita spending. Rwanda has shown the most improvement in Health expenditure per capita, whereby the per capita spending increased exponentially after 2002, reaching a record high of 59 USD in 2014, and it has kept on increasing. Rwanda has surpassed both India and Bangladesh in Government Commitment of Budget to health sector with the record high of 16 percent commitment in 2003 and a whopping 23 percent in 2006, currently standing at around 25 percent. Rwanda has also shown a somehow steady rise in adult female literacy rate, going up from 37 percent in 1991 to around 67 percent according to the latest data, which is appreciable but more needs to be done here. In infrastructure development, Rwandan progress has been steady, boasting good numbers for public access to healthcare facilities and sanitation facilities as compared to India and Bangladesh with a little improvement needed in the sector of training healthcare professionals and caregivers during pregnancy and childbirth. A good explanation of these phenomena can be attributed to the health and Medicare aid provided to Rwanda from external sources and other countries, which currently fund 53 percent of all healthcare resources of Rwanda, which is bringing about major changes in the way things are shaping up. We believe that Rwanda is firmly progressing upon its path to a decreasing MMR and provision of quality healthcare, and the changes are appreciable as seen through the indicators.

The article "Factors That Affect Maternal Mortality in Rwanda: A Comparative Study with India and Bangladesh" was retracted in 2023. Reasons: signs of a paper mill; suspected computer-generated content; unreliable results or conclusions; lack of ethics approval or compliance.

The current healthcare system of Rwanda has been a revelation, whereby the populace is now getting more healthcare coverage in affordable prices. More studies need to be done in the healthcare sector to build upon this good work, which shall help fortify Rwanda reputation not only among sub-Sahara but also Africa as a good example to follow in healthcare delivery. It is believed that this study has a direct impact on the Rwandan maternal healthcare system and it was conducted so that some indicators in the Rwandan healthcare industry may be highlighted and reasons for some shortcomings are investigated. A policy recommendation could be that the Rwandan government and the healthcare sector should take relevant measures that enhance healthcare system, and this ultimately will reduce maternal mortality. This study shows how pivotal the prescribed indicators are when studying the MMR. We can conclude from this study that increase in per capita healthcare expenditure is the most effective element to diminish MMR, followed by numbers of nurses and midwives, budget committed to health, female literacy, and sanitation conditions finally. GDP was not found to have a significant relationship with MMR. More detailed studies may also be conducted to further this idea or to conduct this research in a different way. The idea of this study can be duplicated and can also act as a roadmap for other studies in healthcare provision in Africa and other continents.

The article "Factors That Affect Maternal Mortality in Rwanda: A Comparative Study with India and Bangladesh" was retracted in 2023. Reasons: signs of a paper mill; suspected computer-generated content; unreliable results or conclusions; lack of ethics approval or compliance.

## Figures and Tables

**Figure 1:** Maternal mortality rate.

**Figure 2:** GDP per capita.

**Figure 3:** Health expenditure.

**Figure 4:** Government commitment (monetary).

**Figure 5:** Female literacy rate.

**Figure 6:** Number of hospital beds per 1000 people.

**Figure 7:** Sanitation facilities.

**Figure 8:** Number of nurses and midwives.

**Table 1:** Reports the results of the estimation of multiple regression model (equation (1)) using time series data. The dependent variable is the maternal mortality rate (MMR). Standard errors are reported in italics, and ∗∗∗, ∗∗, and∗ denote statistical significance at the 0.1%, 1%, and 5% levels, respectively. The values in parentheses are *P* values generated from statistical software (R studio).

Dependent variable: maternal mortality rate (MMR)						
	*(1)*	*(2)*	*(3)*	*(4)*	*(5)*	*(6)*
*GDP*	*-1.6990 (0.07332)*					
*FLR*		−0.3497^∗^*(0.02700)*				
*BCH*			−0.5035^∗∗^*(0.005258)*			
*Per capita Health Expenditure*				−17.01^∗∗^*(0.006297)*		
*Nurses and midwives*					−1.8085^∗^*(0.01181)*	
*Sanitation Facilities*						−0.21557^∗^*(0.031)*
*Constant*	1268.18^∗∗^*(0.00855)*	753.93^∗∗^*(0.00905)*	1303.02^∗∗∗^*(0.000485)*	1231.12^∗∗∗^*(0.000353)*	691.10^∗∗^*(0.00153)*	200.69^∗^*(0.0182)*
*R Squared*	*0.5928*	*0.7442*	*0.884*	*0.8733*	*0.8279*	*0.9976*

GDP: gross domestic product; FLR: female literacy rate; BCH: budget committed to health.

## Data Availability

The empirical data used to support the findings of this study is currently under embargo while the research findings are commercialized. Requests for data, 6/12 months after the publication of this article, will be considered by the corresponding author.
